The article "Mechanism of RNA circHIPK3 Involved in Resistance of Lung Cancer Cells to Gefitinib" was retracted in 2024. Reasons: signs of a paper mill; suspected computer-generated content; unreliable results or conclusions; concerns about the data.

# Mechanism of RNA circHIPK3 Involved in Resistance of Lung Cancer Cells to Gefitinib

**DOI:** 10.1155/2022/4541918

**Published:** 2022-04-19

**Authors:** Yi Zhao, Caiming Zhang, Haibo Tang, Xiaomin Wu, Qiugan Qi

**Affiliations:** Department of Cancer Center, Integrated Hospital of Traditional Chinese Medicine, Southern Medical University, Guangzhou 510315, China

## Abstract

To study the mechanism of circular ribonucleic acid (RNA) circHIPK3 involved in the resistance of lung cancer cells to gefitinib, 110 patients with lung cancer were recruited as the research objects, and the tumor tissue and para-cancerous tissue of each patient's surgical specimens were collected and paraffinized to detect the expression of circHIPK3 in different tissues. Gefitinib drug-resistant cell line of lung cancer was constructed with gefitinib to detect cell apoptosis under different conditions. As a result, the relative expression of circHIPK3 in patients with tumor diameter no less than 3 cm was dramatically inferior to that in patients with tumor diameter less than 3 cm (*P* < 0.05). The relative expression of circHIPK3 in patients with TNM stage II/III was dramatically inferior to that in patients with tumor, node, and metastasis (TNM) stage I (*P* < 0.05). Expression of circHIPK3 in patients with lymph node metastasis was dramatically inferior to that in patients without lymph node metastasis (*P* < 0.05). Of the lung cancer tissues of patients with different TNM stages, only six patients had high expression, and the remaining 104 patients had low expression. Moreover, electrophoresis revealed that circHIPK3 can only be amplified in cDNA, but not in gDNA. Gefitinib-mediated apoptosis rate of lung cancer drug-resistant cell lines decreased notably. In summary, the circular RNA circHIPK3 may have a notably low expression in lung cancer tissues, whose low expression had a certain enhancement effect on the drug resistance of lung adenocarcinoma cells to gefitinib.

## 1. Introduction

Lung cancer is a malignant tumor, mainly originated from the mucosal epithelium of the bronchus, which is classified into small cell carcinoma and nonsmall cell carcinoma according to the histological changes. In recent years, with the serious air pollution and the gradual deterioration of the environment, the global mortality rate of lung cancer is on the rise, seriously threatening people's health [1]. According to the report, global cancer statistics in 2018 showed that lung cancer is the malignant tumor with the highest morbidity and mortality. The incidence of lung cancer in China accounts for one-third of the total, and it is increasing [2]. Some workers in special work environments have been exposed to polycyclic aromatic hydrocarbons for long periods of time. Incomplete combustion of these mixed pollutants at 400-800°C produces benzopyrene and 1, 7-dimethylbenzanthracene. These substances can be inhaled and further oxidized to produce free radicals and lipid peroxides that act on the membrane and endoplasmic reticulum of unsaturated fatty acids, and then peroxidation leads to cell membrane damage. Cells with damaged cell membrane will mutate into cancerous cells, leading to the occurrence of cancer [3, 4]. Data from national Cancer Center showed that in 2020, the number of new lung cancer cases in China would reach 816,000, accounting for 17.9% of all cancers [5]. That is an average of 16 people getting sick every 10 minutes. 719,000 deaths occurred, accounting for 23.8% of all cancers [6]. Gefitinib (Iressa) is an oral epidermal growth factor receptor tyrosine kinase inhibitor (EGFR-TKI), a small molecule compound. It is the world's first marketed drug for targeted and precise treatment of lung cancer [7]. Inhibition of EGFR-TK can hinder tumor growth, metastasis, and angiogenesis, and increase tumor cell apoptosis. Gefitinib is used to treat patients with metastatic NSCLC (NSCLC) whose tumors have specific types of epidermal growth factor receptor (EGFR) gene mutations [8, 9].

circRNA is a new type of RNA molecule that is characterized by a covalent closed loop and widely exists in eukaryotes [10]. circRNA is derived from the exon or intron regions of genes and is abundant in mammalian cells. Studies found that most circRNAs are conserved among different species [11, 12]. Because of its ring structure, it can resist the degradation of RNase R, which is relatively stable [13]. circRNA has attracted more and more attention due to its specificity of expression and complexity of regulation, as well as its important role in disease occurrence [14, 15]. Just like miRNA and long noncoding RNA, circRNA has become a new research hotspot in the RNA field [16]. Since circRNA is usually produced by special variable splicing, more than 80% of circRNAs contain protein-encoding exons, have many identical sequences with homologous mRNAs, can be ceRNAs with each other, and act as sponges to adsorb microRNAs [17, 18]. The circular RNA HIPK3 (circHOPK3) is highly expressed in the liver, brain, and lung, mainly originating from the second exon of the gene HIPK3 [19, 20].

The article "Mechanism of RNA circHIPK3 Involved in Resistance of Lung Cancer Cells to Gefitinib" was retracted in 2024. Reasons: signs of a paper mill; suspected computer-generated content; unreliable results or conclusions; concerns about the data.

In recent years, related studies found that using siRNA to knockdown circHIPK3 can inhibit cell proliferation. In addition, circHIPK3 can adsorb miR-124 in liver cancer and promote the proliferation of liver cancer cells by regulating the expression of target genes. However, its regulation and expression mechanism in lung cancer is still unclear. Therefore, this study was developed to explore the mechanism of the circular RNA circHIPK3 involved in the resistance of lung cancer cells to gefitinib.

## 2. Materials and Methods

### 2.1. Sample Collection

In this study, 110 lung cancer patients admitted to X Hospital from September 2019 to September 2020 were collected as the research objects. Paraffin specimens were collected from 58 male patients and 52 female patients. The study has been approved by the Medical Ethics Committee. Patients and their families understood the study content and methods of specimen acquisition and agreed to sign corresponding informed consent forms.

Inclusion criteria: (i) patients diagnosed with lung cancer by pathology and imaging; (ii) patients aged between 45 and 75 years; (iii) there was no metastasis of lung lesions, mediastinal lymph node enlargement, or pleural hypertrophy; (iv) patients who were not recently treated with other drugs or antibiotics in the study; (v) patients with normal coagulation function and platelets.

Exclusion criteria: (i) patients with diseases of other systems or organs; (ii) patients who had not received cooperative treatment due to personal or other factors; (iii) patients with incomplete clinical data and history information (tumor size, clinicopathological stage (TNM), etc.).

Paraffin sections of tumor tissue and para-cancer tissue (normal lung tissue no less than 5 cm from tumor edge and confirmed by pathological examination) from surgical specimens of each included subject were collected. The collected paraffin samples were sliced with uniform thickness (10 *μ*m/slice) and stored in an enzyme-free centrifuge tube (Shanghai Macklin Biochemical Technology Co., Ltd.) containing xylene (Yantai Ruiteng Intelligent Technology Co., Ltd.).

### 2.2. RNA Extraction from Lung Cancer Tissue Sections

Sectioning: the collected paraffin specimens were sectionalized with a thickness of 10 *μ*m/slice and placed quickly in a 1.5 mL tube. Dewaxing: 1,200 *μ*L xylene was added, shaken quickly to mix, centrifuged at 8,600 rpm for 10 min, which was repeated three times, then supernatant was discarded. The lower layer was added with 1,200 *μ*L anhydrous ethanol, mixed by shaking, centrifuged at 8,600 rpm for 5 min at room temperature, and repeated twice. The supernatant was discarded, and the lower layer was dried in an oven at 37°C for half an hour. Then, 200 *μ*L lysate and 5 *μ*L Proteinase K (20 mg/mL) were added. After the tissue was dissolved, it was bathed in water at 95°C for 10 min and centrifuged at 8,600 rpm at room temperature for 5 min. The supernatant was absorbed and transferred to a new Rnase-free centrifuge tube. 220 *μ*L buffer RB was added, shaken, and mixed, then added with anhydrous ethanol, and mixed again.

700 *μ*L solution and precipitate were absorbed and added to the adsorption column, centrifuged at high speed for 1 min. The waste solution was filtered and repeated several times until the solution and precipitate passed through the adsorption column. 80 *μ*L DNase I working solution was added to the center of the adsorption column and left for 15 min at room temperature. 500 *μ*L protein-free RW1 was added and centrifuged, then added with rinse solution, centrifuged again, and the waste solution was discarded. After drying, the adsorption column was transferred to a new RNase-free centrifuge tube. 35 *μ*L RNase-free ddH_2_O was added and centrifuged at 8,600 rpm for 5 min to obtain RNA solution. RNase R was used to process the extracted total RNA to avoid artifacts. RNase R processing reaction system: 2 *μ*g RNA, 1 *μ*L RiboLock, 2 *μ*L 10x RNase R reaction buffer, and 1 *μ*L RNase R, with sterile water supplementing the system to 20 *μ*L [21]. The instructions were followed, and random primers were used for reverse transcription to synthesize cDNA. 2 *μ*L 5 × PrimeScript Buffer, 0.5 *μ*L enzyme mix I, 0.5 *μ*L random 6 mers, and 7 *μ*L total RNA were added to a 0.2 mL enzyme-free EP tube to configure a 10 *μ*L system. The EP tube was closed and shaken for 15 s to mix, centrifuged, and put in the reverse transcription machine. The reverse transcription conditions: 37°C for 15 min, 85°C for 5 sec. After the reaction, the synthesized cDNA was transferred to -20°C refrigerator for storage. The length of circHIPK3 searched on NCBI was 1,099 bp, and the specific base sequence was as follows: GTATGGCCTCACAAGTCTTGGTCTACCCACCATATGTTTATCAAACTCAGTCAAGTGCCTTTTGTAGTGTGAAGAAACTCAAAGTAGAGCCAAGCAGTTGTGTATTCCAGGAAAGAAACTATCCACGGACCTATGTGAATGGTAGAAACTTTGGAAATTCTCATCCTCCCACTAAGGGTAGTGCTTTTCAGACAAAGATACCATTTAATAGACCTCGAGGACACAACTTTTCATTGCGACAAGTGCTGTTGTTTTGAAAAACACTGCAGGTGCTACAAAGGTCATAGCAGCTCAGGCACAGCAAGCTCACGTGCAGGCACCTCAGATTGGGGCGTGGCGAAACAGATTGCATTTCCTAGAAGGCCCCCAGCGATGTGGATTGAAGCGCAAGAGTGAGGAGTTGGATAATCATAGCAGCGCAATGCAGATTGTCGATGAATTGTCCATACTTCCTGCAATGTTGCAAACCAACATGGGAAATCCAGTGACAGTTGTGACAGCTACCACAGGATCAAAACAGAATTGTACCACTGGAGAAGGTGACTATCAGTTAGTACAGCATGAAGTCTTATGCTCCATGAAAAATACTTACGAAGTCCTTGATTTTCTTGGTCGAGGCACGTTTGGCCAGGTAGTTAAATGCTGGAAAAGAGGGACAAATGAAATTGTAGCAATCAAAATTTTGAAGAATCATCCTTCTTATGCCCGTCAAGGTCAAATAGAAGTGAGCATATTAGCAAGGCTCAGTACTGAAAATGCTGATGAATATAACTTTGTACGAGCTTATGAATGCTTTCAGCACCGTAACCATACTTGTTTAGTCTTTGAGATGCTGGAACAAAACTTGTATGACTTTCTGAAACAAAATAAATTTAGTCCCCTGCCACTAAAAGTGATTCGGCCCATTCTTCAACAAGTGGCCACTGCACTGAAAAAATTGAAAAGTCTTGGTTTAATTCATGCTGATCTCAAGCCAGAGAATATTATGTTGGTGGATCCTGTTCGGCAGCCTTACAGGGTTAAAGTAATAGACTTTGGGTCGGCCAGTCATGTATCAAAGACTGTTTGT TCAACATATCTACAATCTCGGTACTACAG.

The article "Mechanism of RNA circHIPK3 Involved in Resistance of Lung Cancer Cells to Gefitinib" was retracted in 2024. Reasons: signs of a paper mill; suspected computer-generated content; unreliable results or conclusions; concerns about the data.

The designed upstream and downstream primers were as follows: circHIPK3-F: TAGACTTTGGGTCGGCCAGT; circHIPK3-R: TGGAATACACAACTGCTTGGC.

The expression of circHIPK3 was detected by real-time fluorescence quantitative polymerase chain reaction (PCR). circHIPK3 is derived from the HIPK3 gene and consists of exon 2 (1,099 bp) head-to-tail splicing. Head-to-tail splicing can be generated by trans-splicing or genome rearrangement. The sequence is a circular sequence, which is assembled from the first position of the corresponding linear RNA, and a new unique sequence is generated at the reverse splicing site. The circRNA specific primers were designed with this as the target sequence, so as to specifically recognize circRNA and distinguish circular sequence from linear RNA. The identification and location of circHIPK3 was shown in Figure 1.

### 2.3. Cell Culture and Passage

Serum-free cell freezing medium (RPMI) 1640 cell culture medium consisted of 10% fetal bovine serum (FBS) (Gibco BRL, USA), 100 U/mL penicillin (Hubei Yangxin Pharmaceutical Technology Co., Ltd.) and 100 mg/mL streptomycin (Shanghai Yuanye Biological Technology Co., Ltd.). The cell cryopreservation tube was taken out of the liquid nitrogen and quickly melted in a constant temperature water bath at 37°C. The thawed cell cryopreservation solution was transferred to a centrifuge tube containing cell culture medium and centrifuged at high speed for 5 min. Then, after cell culture medium was added to the lower sediment to resuspend the cells, they were transferred to RPMI medium and incubated at constant temperature. The medium was changed once the cells grew adherently.

After the cell coverage in the culture dish reached more than 80%, passaging began. After the cell culture solution was aspirated, trypsin digestion solution was added, and cells were observed under a microscope. After culturing until the cells became round, culture medium was added to stop the digestion, and the cells were resuspended and passed to a culture dish.

### 2.4. Construction of Gefitinib-Resistant Cell Lines

Gefitinib was dissolved in dimethyl sulfoxide (DMSO) (Abis (Shanghai) Biotechnology Co., Ltd.). The methyl tetrazolium (MTT) assay was used to determine the median lethal concentration of gefitinib on lung cancer cells (the concentration of the poison that caused half of the tested animals or cells to die in an acute toxicity test). In this study, human lung adenocarcinoma cell line A549 was used to induce gefitinib-resistant cell lines. Resistant cells were induced by a combination of high-dose shocks and gradually increased doses. MTT assay was used to determine the 50% inhibitory concentration (IC_50_) of gefitinib on sensitive cells was 1.78 mol/L. Then, the culture medium containing 17.5 *μ*mol/L gefitinib was used for 24 h, and the medium containing half of the inhibitory concentration gefitinib was immediately replaced for 5-10 d, until the cells grew steadily and were subcultured for 3 times. IC_50_ was determined again. The medium containing 17.5 *μ*mol/L gefitinib was cultured for 24 h, and the medium with gradually increased inhibitory concentration of gefitinib was replaced until the cells grew statically in the medium containing 17.5 *μ*mol/L gefitinib and were continuously passed for 3 times. Then, the IC_50_ of gefitinib was 34.5 *μ*mol/L and was named A549/GR.

The article "Mechanism of RNA circHIPK3 Involved in Resistance of Lung Cancer Cells to Gefitinib" was retracted in 2024. Reasons: signs of a paper mill; suspected computer-generated content; unreliable results or conclusions; concerns about the data.

### 2.5. MTT Colorimetric Detection

Single cell suspension was prepared with culture medium containing 10% fetal bovine serum and inoculated into 96-well plates with 1,000-10,000 cells per well, and volume of each well was 200 *μ*L. The cells were routinely cultured for 3 to 5 days, 20 *μ*L of MTT solution (5 mg/mL, prepared by PBS) was added to each well for 4 h, and the culture was terminated. The supernatant cultured in the hole should be carefully sucked and discarded. For suspended cells, the supernatant should be discarded after centrifugation. 150 *μ*L dimethyl sulfoxide (DMSO) was added to each well and shaken to dissolve completely. At 490 nm, the light absorption value (OD) of each hole was measured by enzyme-linked immunosorbent assay (ELISA) and recorded. The cell growth curve was plotted with time as abscissa and light absorption value as ordinate.

### 2.6. Statistical Methods

SPSS 19.0 was employed for data statistics and analysis. Mean ± standard deviation ($\overset{¯}{x}\pm s$) was how measurement data were expressed, and percentage (%) was how count data were expressed. Analysis of variance was used for pairwise comparison. The difference was statistically considerable with *P* < 0.05.

## 3. Results

### 3.1. circHIPK3 Expression in Different Patients

Figure 2 showed the comparison of the relative expression levels of circHIPK3 in male and female patients and patients of different ages. Among the patients included in the study, there was no considerable difference in the relative expression of circHIPK3 between male patients and female patients (*P* > 0.05). There was also no considerable difference in the relative expression of circHIPK3 between patients less than 60 years old and patients no less than 60 years old (*P* > 0.05).

### 3.2. Expression of circHIPK3 in Different Tumor Types

Figure 3(a) showed the comparison of the relative expression levels of circHIPK3 in patients with tumor diameters less than 3 cm and tumor diameters no less than 3 cm, as well as patients with tumor T staging of stage I and II/III. The relative expression of circHIPK3 in patients with tumor diameter no less than 3 cm was dramatically inferior to that in patients with tumor diameter less than 3 cm (*P* < 0.05). The relative expression of circHIPK3 in patients with T stage II/III tumors was dramatically inferior to that in patients with T stage I (*P* < 0.05).

The article "Mechanism of RNA circHIPK3 Involved in Resistance of Lung Cancer Cells to Gefitinib" was retracted in 2024. Reasons: signs of a paper mill; suspected computer-generated content; unreliable results or conclusions; concerns about the data.

Figure 3(b) showed the comparison of the relative expression levels of circHIPK3 in patients with lung cancer patients whose TNM staging was stage I and stage II/III, as well as those with and without lymph node metastasis. The relative expression of circHIPK3 in patients with TNM stage II/III was dramatically inferior to that in patients with TNM stage I (*P* < 0.05). The relative expression of circHIPK3 in patients with lymph node metastasis was dramatically inferior to that in patients without lymph node metastasis (*P* < 0.05).

### 3.3. Expression of circHIPK3 in Different Tumor Types

The circular RNA circHIPK3 is widely and highly expressed in lung cancer cells, mainly located in the cytoplasm, but also in the nucleus. The expression of circHIPK3 in cancer tissues and normal lung tissues adjacent to cancer is notably different, so it is used for the diagnosis of lung cancer. With pathological and imaging findings as diagnostic criteria, Figure 4 showed the receiver operating characteristic (ROC) curve drawn from the diagnosis of lung cancer through circHIPK3. circHIPK3 had high sensitivity and specificity for the diagnosis of lung cancer, can identify tumor tissues, and had high diagnostic value.

### 3.4. Relative Expression Analysis of circHIPK3

The 110 lung cancer patients included in this study were graded into stage I, stage II, and stage III according to the TNM staging. Among them, 39 patients were in TNM stage I, 36 were in stage II, and 35 were in stage III.  Figure 5 showed the measurement results of the relative expression of circHIPK3 in lung cancer tissues of patients with different TNM stages. Among them, the relative expression level of circHIPK3 (log2) > 0 meant high expression, and log2 < 0 meant low expression [22]. Among the lung cancer tissues of patients with different TNM stages, only 6 patients had high expression, and the remaining 104 patients had low expression.

### 3.5. circHIPK3 Amplification and Electrophoresis

The circular RNA circHIPK3 was amplified by designing primers and then electrophoresed on agarose gel plate to get the electrophoresis, as shown in Figure 6. circHIPK3 can only be amplified in cDNA, but not in gDNA.

The article "Mechanism of RNA circHIPK3 Involved in Resistance of Lung Cancer Cells to Gefitinib" was retracted in 2024. Reasons: signs of a paper mill; suspected computer-generated content; unreliable results or conclusions; concerns about the data.

### 3.6. Analysis of Histopathological Characteristics of Lung Cancer

Figure 7 was a microscopic image of the tumor tissue of a lung cancer patient. There was inflammatory interstitial thickening, edema, fibrosis, and partial alveolar collapse. Tumor cells extended along the alveolar wall, and atypical alveolar wall cubic cells extended along the thickened alveolar interval. Focal fibers were accompanied by atelectasis, and inflammatory cell infiltration was seen.

### 3.7. Fluorescence Staining of Lung Cancer Cells

Figure 8 was a fluorescent staining microscopic image of the constructed gefitinib drug-resistant lung cancer cell line. The apoptotic body cells marked in red also included dividing cells (the nucleus had been separated but the two cells had not been completely separated) and cells containing apoptotic bodies. At 200 multiples, there were many circular or other shaped intact stained bodies.

### 3.8. Apoptosis Detection

The surface of normal cells is composed of lipids distributed asymmetrically on the inner and outer lobes of the plasma membrane. Phosphatidylserine is mostly distributed in the inner lobes of the plasma membrane and exposed to the cytoplasm [23]. However, in the process of apoptosis, lipid asymmetry disappears, and phosphatidylserine is exposed on the outer lobules of the plasma membrane. Annexin V is a 36 KDa calcium-dependent phospholipid-binding protein that can bind to phosphatidylserine [24]. Therefore, the fluorescently labeled Annexin V can be used to detect phosphatidylserine exposed to the outside of early apoptotic cells, and it can also stain necrotic cells (midlate apoptotic cells). By costaining with propidium iodide (PI), apoptotic cells were distinguished from necrotic cells.  Figure 9 showed the results of flow cytometry. The upper right quadrant was the midlate apoptotic cells, and the lower right quadrant was the early apoptotic cells. Gefitinib-mediated apoptosis rate of lung cancer drug-resistant cell lines decreased notably.

## 4. Discussion

Gefitinib can specifically block a certain pathway of lung cancer cells, block the conduction, infiltration, and metastasis of lung cancer cells, locate and kill cancer cells, and cause little damage to normal human cells [25, 26]. It is mainly used to treat locally advanced or metastatic NSCLC that is sensitive to EGFR gene. Local NSCLC that has received chemotherapy before can also be used, but the EGFR gene must be tested before using the drug [27]. Wang et al. (2019) [28] first used AGO2 immunopurification to analyze the possibility of circHIPK3 binding to microRNA. AGO2 is the core component of RISC, connecting miRNAs and their mRNA target sites. Therefore, immunopurification of AGO2 under suitable conditions can obtain miRNA and mRNA that bind to each other, thereby identifying the target site of miRNA. Immunofluorescence can also be performed to detect the intracellular localization of the three complexes. Luciferase reporter gene experiment was combined with PCR for verification. The results showed that circHIPK3-related microRNAs can indeed resist luciferase activity, so there was an interaction between microRNAs and circHIPK3. Zhang et al. (2020) [29] identified 71 differentially expressed circRNAs in osteoarthritis and normal cartilage tissues. Coexpression analysis of circRNA and mRNA combined with transcriptome data was implemented to predict their interaction relationship. It was found that the expression of circRNA and interleukin-1 and tumor necrosis factor increased simultaneously. In addition, it was found that circRNA was involved in the degradation of extracellular matrix, and circRNA played an important regulatory role in human cells.

The article "Mechanism of RNA circHIPK3 Involved in Resistance of Lung Cancer Cells to Gefitinib" was retracted in 2024. Reasons: signs of a paper mill; suspected computer-generated content; unreliable results or conclusions; concerns about the data.

In this study, the tumor tissues and para-cancerous tissues from surgical specimens of 110 study subjects were collected to detect differences in the expression of circHIPK3 in different tissues. Moreover, a lung cancer gefitinib drug-resistant cell line was constructed, and cell apoptosis was detected under different conditions, to study the mechanism of circRNA involved in the resistance of lung cancer cells to gefitinib. As a result, the relative expression of circHIPK3 in patients with tumor diameter no less than 3 cm was dramatically inferior to that in patients with tumor diameter less than 3 cm (*P* < 0.05). The relative expression of circHIPK3 in patients with TNM stage II/III was dramatically inferior to that in patients with TNM stage I (*P* < 0.05). In addition, the relative expression of circHIPK3 in patients with lymph node metastasis was dramatically inferior to that in patients without lymph node metastasis (*P* < 0.05). The results indicated that the relative expression of circHIPK3 in the tumor tissues of patients with lung cancer was closely related to the diameter of the patient's tumor, the TNM stage, and the occurrence of lymph node metastasis. However, there was no high correlation with the patient's age, gender, and other information. Among lung cancer tissues of patients with different TNM stages, only 6 patients had high expression, and the remaining 104 patients had low expression. Therefore, circHIPK3 may have a notably low expression in lung cancer tissues and related cell lines, which had a high correlation with the tumor stage of patients. Flow cytometry apoptosis detection results found that gefitinib-mediated apoptosis rate of lung cancer drug-resistant cell lines decreased notably, which was similar to Zhou et al.'s (2020) [30] research, indicating that circHIPK3 had a certain effect on the drug resistance of lung adenocarcinoma cells gefitinib and can enhance its drug resistance.

The article "Mechanism of RNA circHIPK3 Involved in Resistance of Lung Cancer Cells to Gefitinib" was retracted in 2024. Reasons: signs of a paper mill; suspected computer-generated content; unreliable results or conclusions; concerns about the data.

## 5. Conclusion

In this study, tumor tissues and adjacent tissues were collected from surgical specimens of lung cancer patients to detect differences in the expression of circHIPK3 in different patients and different tumor tissues. In addition, a lung cancer gefitinib drug-resistant cell line was constructed to detect cell apoptosis under different conditions. The results showed that the circular RNA circHIPK3 may have a considerably low expression in lung cancer tissues, and its low expression had a certain enhancement effect on the drug resistance of lung adenocarcinoma cells to gefitinib. However, the sample size selected in this study is small, and the representativeness is low. Therefore, the selection of test sample size will be increased in subsequent experiments. Further study is required to clarify the mechanism of circRNA involved in the resistance of lung cancer cells to gefitinib. In short, this study provides a certain theoretical basis and data support for the drug treatment of lung cancer.

## Figures and Tables

**Figure 1:** circHIPK3 reverse splicing site sequence.

**Figure 2:** The expression of circHIPK3 in different lung cancer patients.

**Figure 3:** The expression of circHIPK3 in different tumor types. Note: (a) was tumor size and T stage; (b) was TNM stage and lymph node metastasis. ∗ indicated that the difference was considerable (*P* < 0.05).

**Figure 4:** ROC curve of circHIPK3 for the diagnosis of lung cancer.

**Figure 5:** Relative expression analysis of circHIPK3 in patients with different stages of lung cancer. Note: (a) was TNM stage I; (b) was TNM stage I; (c) was TNM stage III.

**Figure 6:** circHIPK3 electrophoresis diagram.

**Figure 7:** Histopathological characteristics of lung cancer. Note: (a)–(c) were 40× images; (d)–(f) were 100× images.

**Figure 8:** Fluorescent staining microscopic image of the constructed gefitinib drug-resistant lung cancer cell line A549/GR. Note: the multiples of (a)–(d) were 200×; the multiples of (e)–(h) were 200×.

**Figure 9:** Apoptosis results of gefitinib-resistant lung cancer cell line A549.

## Data Availability

The data used to support the findings of this study are included within the article.
